RETRACTED

# Long-Term Outcomes of Endoscopic Intervention in the Treatment of Symptomatic Pancreas Divisum

**DOI:** 10.1155/2022/8508943

**Published:** 2022-04-16

**Authors:** Guanjun Zhang, Shengxin Chen, Daya Zhang, Lang Wu, Mingyang Li

**Affiliations:** Department of Gastroenterology and Hepatology, The First Medical Center of PLA General Hospital, Beijing 100853, China

## Abstract

To evaluate the efficacy and safety of endoscopic retrograde cholangiopancreatography (ERCP) in the treatment of patients with symptomatic pancreas divisum (PD) and to discuss the possible risk factors of endoscopic reintervention for symptomatic PD. A total of 50 patients with symptomatic PD who underwent ERCP from January 2010 to December 2019 were finally brought into study. All patients were divided into the nonage and the adult group according to their ages. Meanwhile, all patients were also divided into the intervention and the reintervention group according to times of ERCP. The long-term outcome of each patient was collected during the follow-up by phone call. The total success rate of ERCP was 94.7% (89/93), and the effective rate of first ERCP was 58% (29/50). There were no statistical differences on the outcomes of ERCP treatment between the adult and nonage group. There were 17 patients with complete pancreas divisum and 19 patients with chronic pancreatitis in the reintervention group, which were more than 6 patients and 8 patients in the intervention group (*P* < 0.05). In bivariate regression analysis, chronic pancreatitis and complete pancreas divisum might be significant risk factors for endoscopic reintervention for patients with symptomatic PD (OR, 8.010, 95% CI, 1.483–43.276, *P*=0.016; OR, 8.869, 95% CI, 1.450–54.254, *P*=0.018, respectively). ERCP in treating adult and nonage patients with symptomatic PD are effective and safe. But, many patients may need endoscopic reintervention. Complete pancreas divisum and chronic pancreatitis may be risk factors of ERCP reintervention for patients with symptomatic PD.

## 1. Introduction

Pancreas divisum (PD), whose morbidity is reported to be less than 10%, is the most common in the congenital anomaly of the pancreas [1]. But among patients with pancreatitis, the prevalence of PD can even reach up to 25% [1, 2]. It is usually asymptomatic, and only a few people may have abdominal pain, acute pancreatitis (AP), and recurrent acute pancreatitis (RAP), which severely interfere with the quality of life. In the embryological development, failure of fusion of the dorsal and ventral pancreatic ducts results in PD [3]. According to the communication degree of these two ducts, PD can be divided into two types: complete and incomplete PD. Complete PD means the dorsal and ventral pancreatic duct are entirely separated, while incomplete PD means the two ducts have a deficient communication. Once pancreatic secretion increases, the minor papilla and narrow dorsal duct will cause the inadequate drainage, which leads to abdominal pain or pancreatitis [4, 5].

RETRACTED

Endoscopic retrograde cholangiopancreatography (ERCP) is known to be the gold standard for diagnosing PD and meanwhile can be the effective therapy of PD, including minor papilla endoscopic sphincterotomy (MiES) and endoscopic dorsal duct stent insertion (EDSi), which may contribute to pain relief and slow progress of chronic pancreatitis [6, 7]. Nevertheless, the articles on the efficacy and safety of ERCP in the treatment of symptomatic pancreas divisum are scarce, and the ERCP experience on children's pancreas divisum is limited. So, we conducted a long-term study to evaluate the efficacy and safety of ERCP in treating adult and nonage patients with symptomatic pancreas divisum.

## 2. Material and Methods

### 2.1. Basic Information

Consecutive patients with symptomatic PD who underwent ERCP from January 2010 to December 2019 were brought into study through the search of electronic medical record database.

The patients included in the study must satisfy the following criteria: (1) PD was definitely diagnosed by ERCP, (2) with pancreatic pain and pancreatitis, and (3) relative clinical data could be collected overall. Meanwhile, the exclusion criteria included: (1) diagnostic or therapeutic ERCP was not performed, (2) abdominal pain was not caused by PD, or (3) the relevant clinical data were unavailable.

According to their ages, these patients were divided into two groups: the nonage group (age <18 years) and the adult group (age ≥18 years); according to whether the endoscopic reintervention was performed or not, the patients were also divided into two groups: the intervention group (only received ERCP treatment one time and symptoms relieved) and the reintervention group (received ERCP treatment at least two times). The comparable table consisted of the following data: age, gender, symptoms, accompanying disease, operation details associated with ERCP, hospital stay, and long-term follow-up outcomes. We acquired the patients' outcomes after ERCP by phone, which included whether symptoms relived or ever reoccurred and underwent surgeries or not (Figure 1). The study was approved by the ethics committee of PLA General Hospital, and sighed informed consents were obtained from all patients.

### 2.2. ERCP Procedures

Patients were sedated with intravenous propofol, directed by anesthetists, or with basic anesthesia when patients could not tolerant the general anesthesia. All ERCP procedures were performed with a standard side-viewing duodenoscope (TJF-140F, TJF-160VF or TJF-160F; Olympus America, Melville, NY, USA) by experienced endoscopists. According to the image of pancreatogram by cannulation of the minor papilla and the major papilla, the endoscopists then performed minor papilla endoscopic sphincterotomy (MiES), pancreatic ductal stone extraction, and endoscopic pancreatic duct stent insertion (EDSi) to relieve patients' symptoms. In this study, during the process of pancreatic duct stent insertion, we select one or two plastic stents to ensure the free flow of succus pancreaticus (Figures 2 and 3).

RETRACTED

The outcomes of ERCP treatment included the success rate, the effective rate, and post-ERCP adverse events. The success rate represented the technical success rate of ERCP, which meant ERCP procedures, such as MiES and EDSi, were performed as planned. The effective rate was the ratio of the number of people with pain relief during a long-term follow-up and the total number of patients who received ERCP treatment. In regard to abdominal pain relief, we used four grades: (1) total relief, (2) partial relief, (3) no relief, and (4) more pain. The first and second grade meant effective treatment, while the third and fourth grade suggested noneffective treatment. The post-ERCP adverse events incorporated post-ERCP pancreatitis (PEP), hemorrhage, infection, and perforation. PEP meant that a patient after ERCP had symptoms related with pancreatitis, such as abdominal pain which continued for more than 24 hours, and serum amylase levels more than 3 times of the upper limit of normal value. Infections signified a patient after ERCP had a fever which was higher than 38°C and continued for 24 hours, with the leukocyte count and neutrophilic granulocyte percentage elevated to more than normal value. Perforation was defined as free gas in the enterocoelia by abdominal X-rays. Hemorrhage meant that a patient after ERCP had newly emerging symptoms related to anemia, such as palpitation or dizziness, with the hemoglobin value falling to less than normal value.

### 2.3. Statistical Analysis

The research data were processed and analyzed by Statistical Product and Service Solutions (SPSS) 20.0 (SPSS Inc., Chicago, IL, USA). Nonparametric variables were shown as mean value ± standard deviation (SD) or median and range. Fisher's exact test or *X*^2^ test was used for dichotomous variables, and unpaired *t*-test was used for measurement data. The multiple logistic regression was used to determine the association between endoscopic reintervention and pancreas divisum type, chronic pancreatitis after adjusting for potential confounders. While *P* < 0.05, the difference between two groups was significant.

RETRACTED

## 3. Results

### 3.1. Patients

A total of 53 patients underwent therapeutic ERCP, but 3 patients were excluded from the study due to lack of explicit diagnosis of PD. Thereinto, 40 adult patients and 10 nonage patients received a median follow-up of 60 months (range, 10–120 months), and the demographic details are presented in Table 1. There were 26 patients with abdominal pain, 8 patients with acute pancreatitis, and 16 patients with recurrent pancreatitis. Patients with symptomatic PD were possibly complicated with other pancreaticobiliary diseases. More than one half of patients had pancreaticobiliary diseases. Among them, 3 patients had intraductal papillary mucinous neoplasms (IPMN), 2 patients had pancreatic cysts, 1 patient had duodenal adenoma, and 22 patients had pancreatic duct stones or pancreatic duct strictures.

### 3.2. ERCP Outcomes

Altogether, 93 ERCP procedures were proceeded, and the total success rate was 94.7% (89/93). The reasons for failures of ERCP were recorded in Table 2. All patients felt pain relief after ERCP during the hospital stay. However, quite a few patients had abdominal pain or pancreatitis relapse during follow-up, and the effective rate of first ERCP was 58% (29/50). According to clinical manifestations, together with pancreatograms, 29 patients (58%) were diagnosed as CP at the same time and 23 patients (46%) were diagnosed as complete pancreas divisum. Whatever CP or pancreatic divisum type, there were no differences between the two groups. Endoscopic interventions mainly included MiES in 40 patients, EDSi in 27 patients, bouginage in 10 patients, pancreatic ductal stone extraction in 14 patients, and biliary duct stone extraction in 4 patients. Pancreatic plastic stents were ranged from 5 to 10 Fr in diameter and 5 to 12 cm in length. Endoscopic pancreatic stent insertion was performed through the minor papilla in 29 patients and through the major papilla in 4 patients. Nonetheless, ERCP procedures made no statistical differences in adult and nonage group. The total incidence of post-ERCP complications was 22% (11/50), only including PEP. There was no significant difference in complications between adult and nonage group.

### 3.3. Long-Term Outcomes

During follow-up, we selected the baseline data of 46 patients who underwent first endoscopic intervention successfully in our endoscopic center in detail, which is shown in Table 3. 26 patients (56.5%) had to take endoscopic reintervention, and a total of 68 ERCP procedures, including 23 adults and 3 nonages, 14 males and 12 females, of whom 10 patients received ERCP more than 2 times, while 20 patients had significant relief of symptoms and did not undergo additional endoscopic intervention, including 13 adults and 7 nonages, 8 males and 12 females. These above data made no statistical differences in two groups. Also, there were no significant differences on clinical indications, accompanying with other pancreaticobiliary diseases, chronic pancreatitis, and post-ERCP complications in two groups, so it seemed that endoscopic reintervention was not related with patients' symptoms or other pancreaticobiliary diseases or post-ERCP complications. However, there were 17 patients with complete PD and 19 patients with chronic pancreatitis in the reintervention group, which were more than 6 patients and 8 patients in the intervention group, and the difference had statistical significances. So, complete PD could possibly led to endoscopic reintervention, due to its more radical anatomic variation and sclerosis of pancreatic duct.

RETRACTED

In bivariate regression analysis, complicated with chronic pancreatitis and complete pancreas divisum were likely to be significant risk factors for endoscopic reintervention for patients with symptomatic PD (OR, 8.010, 95% CI, 1.483–43.276, *P*=0.016; OR, 8.869, 95% CI, 1.450–54.254, *P*=0.018, respectively) (shown in Table 4).

## 4. Discussion

Pancreas divisum (PD) is the most common congenital variation of pancreatic ductal development, which is first described by a anatomist—Joseph Hyrtl, and the morbidity of which is reported to be less than 10% [7, 8]. The pathomechanism of PD is failure of fusion of the ventral and dorsal pancreatic duct during the eighth week of the embryonic development, and the Santorini's duct drains all or most of pancreatic fluid through the minor papilla, which may lead to inadequate drainage [9]. Most patients are possibly asymptomatic or only show dilation of the pancreatic ducts in the computed tomography or magnetic resonance imaging. But, some patients with PD can present different symptoms such as abdominal pain, acute pancreatitis (AP), or chronic pancreatitis (CP), even including nonage patients, and the life quality can be badly influenced. ERCP is generally accepted to be the first choice for symptomatic PD, which can free the drainage of pancreatic juice [10]. So far, relevant researches on the treatment of PD are inadequate, and ERCP experience on children's pancreas divisum is limited. So, in our study, we chose patients with symptomatic PD, who had also undergone MiES or/and EDSi to make a long-term follow-up, aiming to evaluate the efficacy and safety of ERCP for children and tried to discover the possible risk factors of ERCP reintervention.

RETRACTED

In our study, nonages with symptomatic PD are not different from adults in the sex proportion and symptoms. When patients were first admitted to our hospital, 52% (26/50) of patients suffered from abdominal pain, 16% (8/50) suffered from acute pancreatitis, and 32% (16/50) had recurrent acute pancreatitis. Meanwhile 58% (29/50) had chronic pancreatitis, and there were 23 patients with CP in the adult group, while 6 patients in the nonage group, but the difference was not statistically significant. So, the risk of developing CP for nonage is similar with adults with PD. A child with PD should also be payed enough attention and be intervened positively by endoscopy.

Endoscopic treatments for PD mainly include minor papilla endoscopic sphincterotomy (MiES), minor papilla endoscopic dilation (MiED), and endoscopic dorsal duct stent insertion (EDSi), which can keep drainage of pancreatic juice unblocked [10, 11]. Our study shows that 34% (17/50) of patients only received MiES, and others received pancreatic stent insertion, and whoever adult or nonage patients, plans of endoscopic treatment were similar, according to cannulation and pancreatography, which were not different from some relative researches [12].

Even all patients in our study got a short or long relief after ERCP. As for postoperative complications, there were 10 adult patients and 1 nonage patient developing mild acute pancreatitis after ERCP. So, nonage patients did not show more risks than adult patients with symptomatic PD who received ERCP. From Table 1, we could find that 26 (52%) patients had other pancreaticobiliary disease, including 3 (6%) patient with IPMN, 2 (4%) patients with pancreatic cyst, 1 (2%) patient with duodenal adenoma, and 22 (44%) patients with pancreatic duct stones or pancreatic duct stricture. Therefore, we discovered a tendency that patients with PD were more likely complicated with other pancreaticobiliary diseases. A few researchers also obtained the same result as ours [13, 14]. Long-term chronic inflammation of pancreas maybe results in CP and possibly promote the development of tumor [14]. But, due to lack of enough sample, we cannot totally exclude this is a coincidence. We need more studies with a large sample size to prove it and try to discover the clear pathomechanism. But, once patients have other pancreaticobiliary diseases, such as pancreatic tumor, we need to evaluate the significance of ERCP, and maybe these patients should be performed surgery immediately.

Recent researches have reported that the response rate of symptom relief in patients with symptomatic pancreas divisum who underwent ERCP therapy was nearly equal to that of those with surgery, and the difference was not statistically significant [13–15]. But, some patients might need additional ERCP, which increased length of hospital stay. Although our research is a retrospective study, we achieved a high phone follow-up rate, providing accurate information whether they received extra endoscopy treatment. We found 56.5% (26/46) of patients required endoscopic reintervention, which was reconcilable with other studies [9, 10]. So, it is meaningful to understand which is a risk factor of endoscopic intervention for patients with symptomatic PD. We could discover the number of patients with complete pancreas divisum and chronic pancreatitis in reintervention group were more than that in intervention group, and by means of regression analysis, chronic pancreatitis and complete pancreas divisum were possibly significant risk factors for endoscopic reintervention (OR, 0.103, 95% CI, 0.015–0.700, *P*=0.020; OR, 0.05, 95% CI, 0.005–0.474, *P*=0.009; respectively). Similarly, a few researchers also drew this conclusion that there was a trend towards a higher rate of reintervention in the CP group [10, 15]. So, whether patients with complete PD and complicated with chronic pancreatitis are liable to undergo endoscopic reintervention or not should be proved by more clinical trails with a large sample or randomized controlled trials.

RETRACTED

Our study has several strengths. First, we achieved a long-term follow up, so as to evaluate the outcomes of ERCP. Second, the explicit inclusion and exclusion criteria and clear definitions for variables involved mitigate ambiguity. Finally, we found ERCP in treating symptomatic PD for adult and nonage patients are effective and safe, and complete PD and chronic pancreatitis may be risk factors of ERCP reintervention through a comprehensive analysis, which suggests clinical treatment and prognosis in the future.

Our study also has a few limitations. First, the sample size of the study is not large enough, but PD is a relatively rare disease, and the sample size is limited by the incidence of PD. Second, the retrospective nature of the study signified the introduction of heterogeneity, including availability of data and time of data collection. Finally, nonrandomization of study population possibly led to selection bias, reducing the significance of outcomes.

Until now, the number of articles related to PD has been nearly 800, and most of them are case reports and retrospective studies, and a small amount are randomized controlled trial only including a small sample [9, 16, 17]. Prospective trials with a large number of sample sizes are still expected.

## 5. Conclusion

In conclusion, ERCP in treating symptomatic PD for adult and nonage patients are effective and safe, without severe adverse events. Patients with PD are more likely to be complicated with other pancreaticobiliary diseases. During a long-term follow-up, more than a half of patients need endoscopic reintervention. Complete pancreas divisum and chronic pancreatitis may be risk factors of ERCP reintervention for patients with symptomatic PD.

RETRACTED

## Figures and Tables

**Figure 1:** The flow chart of grouping.

**Figure 2:** Endoscopic views from a 42-year-old female patient with complete pancreas divisum. (a) Minor papilla endoscopic sphincterotomy, (b) the whole pancreatic duct dilation, and (c) two plastic stents (7Fr-8 cm, 5Fr-6 cm) were placed in the pancreatic duct.

**Figure 3:** Endoscopic views from a 9-year-old female patient with complete pancreas divisum. (a) There are multiple filling defects (red arrow) in the pancreatic duct through pancreatography. (b) The pancreatic duct is filled well by contrast media after removing stones. (c) A plastic stent (7Fr-6 cm) was placed in the pancreatic duct.

**Table 1:** Baseline characteristics of patients in adult group and nonage group.

Index	Adult	Nonage	*P*
Age	46.5 (20–73)	14 (9–17)	
Sex (male/female)	20/20	3/7	0.308
Indications			
Abdominal pain	21	5	0.349
Acute pancreatitis	5	3	
Recurrent pancreatitis	14	2	
Endoscopic treatment			
MiES	16	1	0.156
MiES + EDSi/only EDSi	24	9	
Pancreas divisum type			0.943
Complete pancreas divisum	19	4	
Incomplete pancreas divisum	21	6	
Hospital stay	17.17 ± 8.87 d	14.30 ± 9.09 d	0.366
With other pancreaticobiliary malformation/disease	21	5	1.000
Complication	10	1	0.550
With chronic pancreatitis	23	6	1.000

**Table 2:** Patients who failed to undergo ERCP.

Patient	Age	Pancreas divisum type	Reason	Final treatment
Lu	53	Incomplete	Minor papilla in the diverticula	Minor papilla endoscopic sphincterotomy + ventral pancreatic duct stent insertion
Xiang	56	Complete	First failure to find minor papilla	Minor papilla endoscopic sphincterotomy + dorsal pancreatic duct stent insertion
Zhu	50	Incomplete	Pancreatic duct stricture	Minor papilla endoscopic sphincterotomy
Pei	33	Incomplete	Swollen minor papilla	Minor papilla endoscopic sphincterotomy + dorsal pancreatic duct stent insertion

**Table 3:** Baseline characteristics of patients in reintervention group and intervention group.

Index	Reintervention	Intervention	*P*
Age (adult/nonage)	23/3	13/7	0.121
Sex (male/female)	14/12	8/12	0.351
Indications			
Abdominal pain	14	11	0.872
Acute pancreatitis	4	4	
Recurrent pancreatitis	8	5	
Pancreas divisum type			0.049
Complete pancreas divisum	14	5	
Incomplete pancreas divisum	12	15	
With other pancreaticobiliary malformation/disease	17	9	0.167
Complication	6	5	1.000
With chronic pancreatitis	19	8	0.024

RETRACTED

**Table 4:** Regression analysis of endoscopic reintervention (ERCP at least two times) for patients with symptomatic PD.

Factors	*β*	Wald *χ*^2^	*P*	OR	95% CI
With chronic pancreatitis	2.081	5.844	0.016	8.010	1.483,43.276
Complete pancreas divisum	2.183	5.579	0.018	8.869	1.450,54.254
With other pancreaticobiliary malformation/disease	1.055	1.997	0.158	2.872	0.665,12.410

## Data Availability

The datasets used and analyzed during the current study are available from the corresponding author on reasonable request.
